The article "Mechano growth factor attenuates mechanical overload-induced nucleus pulposus cell apoptosis through inhibiting the p38 MAPK pathway" was retracted in 2024. Reasons: duplicated images; compromised peer review; concerns about the authorship.

# Mechano growth factor attenuates mechanical overload-induced nucleus pulposus cell apoptosis through inhibiting the p38 MAPK pathway

**DOI:** 10.1042/BSR20182462

**Published:** 2019-03-29

**Authors:** Qing Xu, Haolin Fang, Liang Zhao, Cunxin Zhang, Luo Zhang, Baofang Tian

**Affiliations:** 1 Department of Anesthesia Surgery, Jining NO. 1 People’s Hospital, Affiliated Jining NO. 1 People’s Hospital of Jining Medical University, Jining Medical University, Jining 272000, Shandong, China; 2 Department of Emergency Trauma Surgery, Jining NO. 1 People’s Hospital, Affiliated Jining NO. 1 People’s Hospital of Jining Medical University, Jining Medical University, Jining 272000, Shandong, China; 3 Department of Spine Surgery, Jining NO. 1 People’s Hospital, Affiliated Jining NO. 1 People’s Hospital of Jining Medical University, Jining Medical University, Jining 272000, Shandong, China

**Keywords:** apoptosis, intervertebral disc degeneration, mechano growth factor, mechanical overload, nucleus pulposus

## Abstract

Mechanical overload is a risk factor of disc degeneration. It can induce disc degeneration through mediating cell apoptosis. Mechano growth factor (MGF) has been reported to inhibit mechanical overload-induced apoptosis of chondrocytes. The present study is aimed to investigate whether MGF can attenuate mechanical overload-induced nucleus pulposus (NP) cell apoptosis and the possible signaling transduction pathway. Rat NP cells were cultured and subjected to mechanical overload for 7 days. The control NP cells did not experience mechanical load. The exogenous MGF peptide was added into the culture medium to investigate its protective effects. NP cell apoptosis ratio, caspase-3 activity, gene expression of Bcl-2, Bax and caspase-3, protein expression of cleaved caspase-3, cleaved PARP, Bax and Bcl-2 were analyzed to evaluate NP cell apoptosis. In addition, activity of the p38 MAPK pathway was also detected. Compared with the control NP cells, mechanical overload significantly increased NP cell apoptosis and caspase-3 activity, up-regulated gene/protein expression of pro-apoptosis molecules (i.e. Bax, caspase-3, cleaved caspase-3 and cleaved PARP) whereas down-regulated gene/protein expression of anti-apoptosis molecule (i.e. Bcl-2). However, exogenous MGF partly reversed these effects of mechanical overload on NP cell apoptosis. Further results showed that activity of the p38 MAPK pathway of NP cells cultured under mechanical overload was decreased by addition of MGF peptide. In conclusion, MGF is able to attenuate mechanical overload-induced NP cell apoptosis, and the p38 MAPK signaling pathway may be involved in this process. The present study provides that MGF supplementation may be a promising strategy to retard mechanical overload-induced disc degeneration.

## Introduction

Low back pain is the main cause of disability in middle-aged adults. Generally, intervertebral disc (IVD) degeneration is directly or indirectly related with the low back pain [1]. Current treatments including conservative therapy and operation are just effective in alleviating pain symptom but not in biologically retarding disc degeneration [2]. The key bottleneck point is that the pathogenesis of disc degeneration remains unclear to us.

IVDs locate between two adjacent vertebraes [3]. Because the central nucleus pulposus (NP) tissue contains abundant proteoglycan that is characterized as a negative charge-rich protein [4], IVD absorbs mechanical load and allows multi-directional motion of the spine during daily activities. However, increasing evidence has indicated that mechanical compression is an important regulator of disc biology and that high-magnitude mechanical compression promotes disc degeneration [5–9].

During disc degeneration, NP region first exhibits degenerative changes. At the cellular level, NP cell apoptosis is one of the most common features within the degenerative disc tissue [10–12]. Apoptosis is identified as a process of programmed cell death initiated by activation of caspases (i.e. caspase-3, 6 and 7) [13]. In the past several years, NP cell apoptosis is a research focus in the field of disc degeneration. At the initial research phase, Gruber and Hanley [14] first identified apoptotic cells in the degenerative human discs. After that, Rannou et al. [15] demonstrated that human disc degeneration is positively associated with NP cell apoptosis. Therefore, we speculate that cell apoptosis may be a critical cause of the decrease in cellularity within the NP region during disc degeneration.

Mechano growth factor (MGF), also known as insulin-like growth factor 1 Ec (IGF-1Ec), is a splicing variant of IGF-1. According to previous reports, MGF has great potential in repairing skeletal muscle, heart and neuron [16–19]. Moreover, MGF has been proved to inhibit cell apoptosis in myocytes and chondrocytes [20,21]. Importantly, MGF has been reported to attenuate mechanical overload-induced apoptosis of growth plate chondrocytes [21]. As a cartilaginous tissue, NP tissue has some similar characters of cartilage. However, whether MGF can inhibit mechanical overload-induced NP cell apoptosis remains unclear. In the present study, we mainly aimed to investigate whether the exogenous MGF can attenuate mechanical overload-induced NP cell apoptosis.

## Materials and methods

### Ethical statement

All experiment animals were used according to the guidelines of Ethics Committee at Jining No.1 People’s Hospital Affiliated to Jining Medical University [SWFK (LU) 2054-0016].

### NP cell isolation and culture

Thirty-three Sprague–Dawley rats (males and females, 250 g and 6–8 weeks old) were killed by excessive carbon dioxide inhalation. Then, the spinal column (T10-L5) was separated under sterile conditions. Subsequently, the gel-like NP tissue samples were scraped under a dissecting microscope and digested with 0.25% trypsin for 3–6 min on a shaker. After the first centrifugation (1000 r.p.m., 5 min), the tissue pellets were collected and then were digested with 0.2% (w/v) collagenase type II (Sigma–Aldrich, U.S.A.) at 37°C for 4 h. Thereafter, NP cells were suspended in DMEM/F12 medium containing 10% fetal bovine serum (FBS, Gibco, U.S.A.) in a humid CO_2_ incubator.

To apply the mechanical compression to NP cells *in vitro*, NP cells were seeded onto the cylindric small intestinal submucosa (SIS) cryogel scaffolds (4 × 10^6^ per scaffold). After the NP cells seeded onto the SIS crygel were pre-cultured for 24 h, they were experienced dynamic compression once per day for a total of 7 days using a mechanical compression application machine. To investigate the protective effects of MGF against mechanical compression-induced NP cell apoptosis, NP cells experienced a compressive magnitude of 25% scaffold axial deformation at a frequency of 1.0 Hz for 6 h per day, and the exogenous MGF peptide (40 ng/ml) was added along with the culture medium. The concentration of MGF was designed according to our own experience. NP cells without dynamic compression were used as controls. The culture medium was refreshed every 3 days.

### Cell apoptosis ratio measurement

After culture, the medium in the culture chamber was collected. And then, the scaffolds were cut into fragments and digested with 0.25% trypsin without EDTA for 40 s at 37°C. Subsequently, the culture medium and the cell suspension were mixed together and centrifuged (1000 r.p.m., 5 min, 4°C) to collect NP cell pellets. After discarding the supernatant, the NP cells were suspended by 195 μl Annexin V-FITC binding buffer, followed by incubation with 5 μl Annexin V-FITC solution and 10 μl propidium iodide (PI) solution for 30 min. Finally, NP cells were subjected to a flow cytometry machine. The apoptotic NP cells were identified as Annexin V positive-stained and PI-negative-stained cells, as well as double positive-stained cells.

### Caspase-3 activity detection

Caspase-3 activity was measured using a caspase-3 activity detection kit (Beyotime, China). Briefly, the SIS scaffolds were washed with phosphate buffer solution (PBS) and cut into fragments after culture. Then, the protein supernatant was collected using the lysis solution in the kit. Then, the protein supernatant, reaction buffer and Ac-DEVD-pNA were mixed and used to perform the chemical reaction at 37°C. After reading the optical density (OD) at a wavelength of 405 nm, caspase-3 activity was calculated and normalized to the total protein.

### Real-time PCR analysis

After culture, the SIS scaffolds were cut into fragments. Then, the total RNA was extracted using TRIzol reagent (Invitrogen, USA) and reverse-transcribed using a First Strand cDNA Synthesis Kit (Roche, Switzerland). Next, real-time PCR was carried out using the SYBR Green Mix (TOYOBO, Tapan) on an Applied Biosystems^®^ 7500 Real-Time PCR System. The PCR cycles conditions were: 3 min at 95°C, followed by 40 amplification cycles of 15 s at 95°C, 15 s at 56°C and 15 s at 72°C. The primers of target genes (Table 1) were designed using the Primer 5.0 Software and synthesize by a domestic company (Sangon Biotech, China). The relative expression of target genes was calculated using the method of 2^−ΔΔ*C*^_t_.

**Table 1:** Primers of target genes

Gene	Forward (5′–3′)	Reverse (5′–3′)
*GAPDH*	ATCAAGAAGGTGGTGAAGCA	AAGGTGGAAGAATGGGAGTTG
*Bax*	TTGCTACAGGGTTTCATCCA	TGTTGTTGTCCAGTTCATCG
*Bcl-2*	GGTGGACAACATCGCTCTG	CAGCCAGGAGAAATCAAACA
*Caspase-3*	ACGGGACTTGGAAAGCATC	TAAGGAAGCCTGGAGCACA

### Western blotting analysis

The SIS scaffolds were cut into fragments and lysed by RIPA buffer (Beyotime, China) with intermittent ultrasound on ice. Then, the total protein supernatant was collected by centrifugation at 1.5 × 10^4^ r.p.m. for 5 min. After protein concentration was measured using a BCA Protein Assay Kit (Beyotime, China), the protein samples were separated by SDS/PAGE and transferred on to the PVDF membranes. Subsequently, the PVDF membranes were incubated with the primary antibodies (β-actin: Abcam, ab8227; cleaved PARP: Abcam, ab32064; cleaved caspase-3: Abcam, ab49822; Bcl-2: Abcam, ab692; Bax: Abcam, ab32503; p38 MAPK: Cell Signaling Technology, #14451; p-p38 MAPK: Cell Signaling Technology, #9216) overnight at 4°C and the secondary antibodies at room temperature for 2 h. Subsequently, cross-reactivity was visualized using the enhanced chemiluminescence Western blotting detection reagents (BeyoECL Plus, beyotime, China). Finally, the protein bands were analyzed by scanning densitometry.

### Statistical analysis

Every experiment was independently performed at least for three-times. Data were expressed as mean ± standard deviation (S.D.). Statistical analysis was performed using one-way analysis of variance (ANOVA). The *post hoc* test was determined by LSD test. A *P*-value <0.05 indicated a statistical significance.

## Results

### Cell apoptosis ratio

Results showed that mechanical overload significantly increased NP cell apoptosis ratio compared with the control group. However, when the MGF peptide was added into the culture medium, NP cell apoptosis ratio was significantly decreased (Figure 1).

**Figure 1:** Nucleus pulposus cell apoptosis ratio analyzed by flow cytometry Data are expressed as mean ± S.D., *n*=3. *: Indicates a significant difference (*P*<0.05).

### Caspase-3 activity

Results showed that caspase-3 activity was significantly increased in the NP cells subjected to mechanical overload. However, when the MGF peptide was added into the culture medium, caspase-3 activity was significantly decreased (Figure 2).

**Figure 2:** Analysis of caspase-3 activity Data are expressed as mean ± S.D., *n*=3. *: Indicates a significant difference (*P*<0.05).

### Analysis on mRNA expression of apoptosis-related molecules

In the present study, gene expression of pro-apoptosis molecules (caspase-3 and Bax) and anti-apoptosis molecule (Bcl-2) was analyzed. Results showed that mechanical overload significantly up-regulated mRNA expression of caspase-3 and Bax, but down-regulated mRNA expression of Bcl-2. On the contrary, MGF peptide partly down-regulated mRNA expression of caspase-3 and Bax, but up-regulated mRNA expression of Bcl-2 in NP cells subjected to mechanical overload (Figure 3).

**Figure 3:** Real-time PCR analysis of apoptosis-related molecules (Bcl-2, Bax and caspase-3) Data are expressed as mean ± S.D., *n*=3. *: Indicates a significant difference (*P*<0.05).

### Analysis on protein expression of apoptosis-related molecules

Similarly, protein expression of apoptosis-related molecules (Bcl-2 and Bax) and apoptosis markers (cleaved caspase-3 and cleaved PARP) was analyzed. Results showed that mechanical overload significantly up-regulated protein expression of cleaved caspase-3, cleaved PARP and Bax, but down-regulated protein expression of Bcl-2. On the contrary, MGF peptide partly down-regulated protein expression of cleaved caspase-3, cleaved PARP and Bax, but up-regulated protein expression of Bcl-2 in NP cells subjected to mechanical overload (Figure 4).

**Figure 4:** Western blot analysis of apoptosis-related molecules (Bcl-2, Bax, cleaved PARP and cleaved caspase-3) Data are expressed as mean ± S.D., *n*=3. *: Indicates a significant difference (*P*<0.05).

### Analysis on the activity of the p38 MAPK pathway

To tentatively investigate whether the p38 MAPK pathway was involved in this process, we detected activity of the p38 MAPK pathway. Results showed that activity of the p38 MAPK pathway was significantly increased in the NP cells subjected to mechanical overload. However, when the MGF peptide was added into the culture medium, activity of the p38 MAPK pathway was significantly decreased (Figure 5).

**Figure 5:** Analysis of activity of the p38 MAPK pathway by Western blot assay Data are expressed as mean ± S.D., *n*=3. *: Indicates a significant difference (*P*<0.05).

## Discussion

IVD is a cartilaginous tissue connecting two adjacent vertebraes which absorb biomechanical loads [3]. The central gelatinous NP is a major component of the disc and largely responsible for its mechanical function [3]. A decrease in the NP cell density caused by cell apoptosis is an important cellular pathology during disc degeneration [11]. As an important initiator of disc degeneration, mechanical overload has been reported to be closely related with disc cell apoptosis and thus contributes to disc degeneration [5,22–24]. Therefore, inhibition of mechanical overload-induced disc cell apoptosis may be a potential treatment of disc degeneration. In the present study, we demonstrated for the first time that exogenous MGF peptide was able to attenuate NP cell apoptosis under mechanical overload and the p38 MAPK pathway was involved in this regulatory process.

Previously, many studies have demonstrated that cellular apoptosis participates in disc degeneration [25–28]. In most cases, apoptosis is identified by the method of terminal deoxynucleotidyl transferase-mediated dUTP nick-end labeling (TUNEL) staining [29–31]. Moreover, a previous study has reported that the IVDs from patients have considerably more TUNEL-positive cells than the healthy control discs [15]. Therefore, there is an association between human disc degeneration and NP cell apoptosis.

During daily activities, the IVDs are subjected to various mechanical loads. Previously, many studies have indicated that mechanical compression is an important regulator of disc cell biology [32–36]. In the present study, we found that mechanical overload significantly increased NP cell apoptosis ratio, caspase-3 activity, up-regulated gene/protein expression of Bax, caspase-3, cleaved caspase-3 and cleaved PARP, whereas down-regulated gene/protein expression of Bcl-2. These findings indicate that mechanical overload contributes to NP cell apoptosis. This is in line with previous studies demonstrating that an excessive mechanical loading induces disc cell death [5,23,24,37].

MGF is an autocrine and endocrine growth factor whose expression is identified in many tissues [18]. MGF is able to regulate cell proliferation, cell differentiation and cell migration, and exhibits some protective effects against different harmful stimuli [38]. However, whether MGF has protective functions against harmful stimuli-induced disc degeneration remains unclear. In the present study, we found for the first time that exogenous MGF peptide significantly decreased cell apoptosis ratio, caspase-3 activity, down-regulated gene/protein expression of Bax, caspase-3, cleaved caspase-3 and cleaved PARP, whereas up-regulated gene/protein expression of Bcl-2 in NP cells under mechanical overload. These results suggest that exogenous MGF peptide is helpful to alleviate mechanical overload-induced NP cell apoptosis. In line with this, several previous studies have also demonstrated that MGF is able to alleviate mechanical load-induced damage in growth plate chondrocytes [21], and to regenerate cartilage tissues [39,40]. However, the molecular mechanisms through which MGF exerts its protective functions against mechanical overload-induced NP cell apoptosis were not fully understood. Here, we tentatively explored activity of the p38 MAPK signaling pathway in this process. We found that mechanical overload significantly increased activity of the p38 MAPk pathway, whereas the exogenous MGF peptide partly decreased activity of the p38 MAPK pathway, indicating that MGF may play its protective role through regulating the p38 MAPK pathway.

The present study has some points need to be explained. First, we just designed one concentration of MGF in the present study. The dose-dependant effects of MGF will be further investigated in the future. Second, an intact disc contains NP, annulus fibrosus and cartilage endplate. The relationship between these three closely connected parts was not studied in the present study. Third, the rat NP tissue contains lots of notochordal cells which are also sensitive to mechanical stimulation. The existence of notochordal cells may bring some unknown effects to the present results.

In a word, we explored the effects of MGF on mechanical overload-induced NP cell apoptosis, and the potential signaling transduction pathway in this process. Our results indicated that MGF could attenuate mechanical overload-induced NP cell apoptosis through regulating the p38 MAPK pathway. The present study implies that MGF supplementation may be a promising strategy to retard mechanical overload-induced disc degeneration.

## Abbreviations

Bax: Bcl-2 Associated X protein
BCA: bicinchoninic acid
Bcl-2: B cell lymphoma/lewkmia-2
IGF-1Ec: insulin-like growth factor 1 Ec
IVD: intervertebral disc
MAPK: mitogen-activated protein kinase
MGF: mechano growth factor
NP: nucleus pulposus
PI: propidium iodide
RIPA: radio-immunoprecipitation assay
SIS: small intestinal submucosa
TUNEL: terminal deoxynucleotidyl transferase-mediated dUTP nick-end labeling
